# Knockdown of lncRNA *HOXD-AS2* Improves the Prognosis of Glioma Patients by Inhibiting the Proliferation and Migration of Glioma Cells

**DOI:** 10.1155/2022/9337647

**Published:** 2022-11-09

**Authors:** Feng Chen, Ru-Ru Zhao, Qian Li, Zhen-Hua Chen, Chun Luo

**Affiliations:** ^1^Department of Neurosurgery, Tongji Hospital, School of Medicine, Tongji University, Shanghai, China; ^2^Shanghai First Maternity and Infant Hospital, Tongji University School of Medicine, Shanghai, China; ^3^Department of Neurosurgery, Affiliated Hospital 2 of Nantong University, Nantong, China

## Abstract

**Objective:**

Increasing studies reported that long noncoding RNAs are involved in regulating glioma progression. However, the specific roles and mechanisms of lncRNAs in glioma remain unclear. Here, we sought to explore the functions of HOXD-AS2 in glioma progression.

**Methods:**

Gene expressions of lncRNAs in 5 normal brain tissue specimens and 5 glioblastoma tissue specimens were detected by gene expression profile chip technology. Bioinformatic analysis was performed to see whether differential expression of lncRNAs played any significant role in glioma occurrence and progression. The relationship between HOXD-AS2 level and clinical prognosis of the patients was analyzed. HOXD-AS2 was specifically interfered with by siRNA technology to observe its effects on U251 cell growth, proliferation, apoptosis, and invasion.

**Results:**

The expression level of HOXD-AS2 gene in glioma was significantly higher than that in the normal brain tissue, which was related to the tumor grade. The level of HOXD-AS2 gene in patients with high-grade glioma was higher than that in patients with low-grade glioma. High expression of HOXD-AS2 gene was a risk factor for poor prognosis of glioma patients. Knocking down the expression of HOXD-AS2 in glioma cell line U251 arrested the cell cycle and reduced the cell proliferation. Furthermore, it could significantly reduce the migration ability of the cells but had no significant effect on the invasion.

**Conclusion:**

HOXD-AS2 is an oncogenic lncRNA associated with the poor prognosis of glioma. Knockdown of *HOXD-AS2* may reduce the growth of glioma, which may provide a new avenue for treatment.

## 1. Introduction

Glioblastoma (GBM) is the most malignant form of primary brain tumor, associated with an extremely poor prognosis [1]. The median survival time of patients with GBM is only 15 months [2]. Although comprehensive treatment based on surgical resection, local radiotherapy, and systematic chemotherapy has been widely used, the prognosis of patients with GBM remains unsatisfactory, and most patients experience relapse within a short time after operation. It is therefore essential to gain a better understanding of the mechanism of tumor occurrence at the genetic and molecular levels for the sake of improving the effectiveness of therapy for glioma.

Long noncoding RNAs (lncRNAs) are a class of RNA with a length of more than 200 bp and no protein-coding ability [3]. Unlike microRNA and other small noncoding RNAs, lncRNAs can regulate downstream target genes through cis- and trans-regulation at transcriptional and posttranscriptional levels [4]. Although many lncRNAs have proved to play a crucial role in human diseases, such as osteosarcoma [5] and bone mass [6], the functions of most lncRNAs in tumors remain unknown. With the development of high-throughput gene sequencing technology, the abnormal expression of some lncRNAs has been found to be closely related to the proliferation, invasion, recurrence, and prognosis of glioma. A well-known lncRNA molecule, *HOTAIR (Hox antisense intergenic RNA)*, the antisense strand of the *Hox* gene, has been widely studied in many tumors. It was initially found to be associated with poor prognosis in multiple malignant tumors, including glioma [7]. Some functional experiments have shown that interference with *HOTAIR* can arrest the cell cycle, slow cell growth, and weaken the invasive ability of glioma cells [8].

Similar to *HOTAIR*, *HOXD-AS2* is located on chromosome 2 and is the antisense chain of *homeobox D* gene. Initially, it was found that *lncRNA HOXD-AS2* could regulate the A172 cell cycle to promote glioma progression [9]. However, a recent study has shown that decreased expression of the long noncoding RNA *HOXD-AS2* promotes gastric cancer progression by targeting *HOXD8*, which activates the *PI3K/Akt* signaling pathway [10]. In our previous study with microarrays of glioma specimens, we found that *HOXD-AS2* was aberrantly expressed in glioma [11]. However, the involvement of *HOXD-AS2* in glioma progression remains unclear.

The purpose of this study was to investigate the relationship between the differential expression of the lncRNA *HOXD-AS2* gene and the pathological grade and malignant behavior of glioma in an attempt to seek new strategies for diagnostic markers and prognostic targets of glioma.

## 2. Materials and Methods

### 2.1. Gene Chip Technology and Target Gene Screening

Five tumor tissue samples were selected from patients with primary GBM, and five normal brain tissue samples were selected from patients who underwent internal decompression and resection after brain trauma with no tumor or other pathological changes. All the patients received treatment in the Department of Neurosurgery at Tongji Hospital (Shanghai, China) from January 2018 to December 2019. The pathological grades and types of the tumors were confirmed by two pathologists, and the study procedures were approved by the Ethics Committee of Tongji Hospital.

Total RNA was extracted from the GBM and normal brain tissues, and differentially expressed lncRNAs in the tumor tissue were screened out using lncRNA high-throughput hybridization on the chip. Sequence alignment analysis was performed using the Basic Local Alignment Search Tool (BLAST). When these findings were combined with the results of bioinformatic analysis, *HOXD-AS2* was determined to be the target gene of this study, because it is highly expressed in tumor tissues. Five genes (*HOXD-AS2, HOXA11-AS, HOXA2, MMP7, and MMP9*) were randomly selected from the microarray data, and their expression in the five GBM tissue samples *vs.* five normal brain tissue samples was detected by real-time quantitative PCR (RT-qPCR). The primer sequences are shown in Table 1. The logarithm of the ratio of gene expression in tumor and normal brain tissues was calculated and compared with the microarray results to verify the accuracy of the microarray data.

### 2.2. Expanded Sample Size Verification and Analysis of Survival Prognosis

According to the World Health Organization classification standard, 102 glioma tissue specimens were taken from patients with grade I glioma (*n* = 8), grade II glioma (*n* = 37), grade III glioma (*n* = 24), and grade IV glioma (*n* = 33), and five normal brain tissue specimens were taken from parts of the brain tissues during internal decompression and resection after traumatic injuries.

Fifteen of the 102 glioma patients were lost to follow-up, and the remaining 87 patients had complete clinical data and prognostic information. Among them, 48 were male and 39 were female, including 52 patients younger than 55 years and 35 patients ≥ 55 years. The tumor size was <5 cm in 30 cases and ≥5 cm in 57 cases. According to the degree of tumor resection during operation, total resection was performed in 52 cases, subtotal resection in 29 cases, and partial resection in 6 cases. The survival time started from the second day after operation to the day of clinical death (or the last follow-up day) of the patient. The follow-up period was 3–47 months. The clinical data were obtained from the patient's medical records according to the patient's hospitalization number. The patients were followed up via telephone interviews.

### 2.3. Establishment of the GBM Cell Model with Interfering Expression of lncRNA

Using the siRNA technique, the expression of *HOXD-AS2* was knocked down to observe the effect on the function of glioma cell line U251 (Cell Bank of the Chinese Academy of Sciences, Shanghai, China) in an experimental group and the control group. The control group was divided into a blank control group (mock, M) and a negative control group (NC). In the experimental group, three siRNAs were designed and synthesized by Shanghai GenePharma: *HOXD-AS2-homo-136, HOXD-AS2-homo-584, and HOXD-AS2-homo-633* (Table 2). Invitrogen Lipofectamine 3000 was used as a vector to transfect glioma cell line U251.

The siRNA was diluted with Opti-MEM, and 125 *μ*l Opti-MEM and 5 *μ*l siRNA solution were added to each tube, gently blown with a 200 *μ*l gun head, and fully mixed to prepare an siRNA premix. The siRNA premix was added to the diluted Lipo 3000, mixed evenly, and allowed to rest for 5 min. The cells in the 6 cm dish were replaced with serum-free medium, and the prepared siRNA-Lipo 3000 complex was aspirated and transferred to the medium. The interference efficiency was measured.

### 2.4. RT-qPCR

RNA was extracted from the pathological tissue samples or cells frozen in liquid nitrogen. The primers were designed across the intron region using Primer Premier 5.0 software and supplemented by the following manual analysis: length of the primer: 18–25 bp; *G* + *C* content: 40%–60%; secondary structure: avoiding primer dimers and hairpin structures; and 3′ ends: strictly paired and 5′ ends modified. *GAPDH* was selected as the internal reference gene.

### 2.5. Detection of Cell Proliferation Ability

Cell proliferation ability was detected using a Cell Counting Kit-8 (CCK-8): 100 *μ*l cell suspension was inoculated into a 96-well plate in the NC group, SiHOXD-AS2-1 experimental group, and SiHOXD-AS2-2 experimental group, with five wells used for each group. Subsequently, 10 *μ*l CCK-8 solution was added to each well containing the seeded cells, making sure that the reagent was added obliquely against the wall of the culture plate to reduce bubble generation. CCK-8 solution was added at 12, 24, 36, and 48 h, and the OD at 450 nm was recorded.

### 2.6. Cell Proliferation Assay

The transfected cells in the six-well plate were cultured for 24 h, washed with PBS, digested with trypsin, and resuspended with 1 ml fresh medium. Cells were labeled with the 5-ethynyl-2-deoxyuridine (EdU) and then fixed and stained.

### 2.7. Cell Cycle Assay

Cells were added to 1 ml 70% ethanol precooled in an ice bath, fixed overnight, and washed with ice-cooled PBS. For the preparation of the propidium iodide (PI) staining solution, each sample contained 0.5 ml staining buffer solution, 25 *μ*l propidium iodide staining solution (20 ×), and 10 *μ*l RNase A (50 ×). The samples were blown gently and mixed well. After adding 500 *μ*l PI for staining, the EP (Eppendorf) tube was sealed with sealing glue and kept in a water bath for 30 min at 37°C, followed by a 4°C refrigerator. Flow cytometry was performed at a slow rate of 100–300 cells per second.

### 2.8. Apoptosis Assay

One microliter of apoptosis-inducing reagent A (Beyotime Biotechnology) was added to each of the three wells of the six-well plate, and the cells were cultured overnight. The cells were resuspended sufficiently with 300 *μ*l of 1 × binding buffer. After the addition of 5 *μ*l Annexin V-FITC, the cells were incubated for 15 min. Subsequently, 10 *μ*l PI was added to each tube, and the cell suspension was incubated for 5 min and measured using a flow cytometer.

### 2.9. Cell Migration Assay

Briefly, a 2.5 *μ*l white gun head was sterilized, placed in the center of a six-well plate, and a scratch was made perpendicular to the plane. After replacement with serum-free medium, the plate was observed and photographed with a microscope, which was recorded as 0 h. Photography was repeated at 12 h of intervals to observe cell crawling on both sides of the scratch and the morphology of the cells. The serum-free medium was replaced every 2–3 days.

### 2.10. Cell Invasion Assay

For this assay, 4 × 10^4^ cells were placed in a chamber. After 24–36 h, the chamber was gently rinsed with preheated PBS solution, and the upper surface cells were scraped off. An additional three wells were supplemented with 1 ml of 4% paraformaldehyde, put into a small chamber, and fixed for 30 min. The chamber was taken out, rinsed with PBS, and air-dried. An additional three wells were supplemented with 1 ml crystal violet staining solution, put into a small chamber, and soaked for 30 min. The chamber was flushed with distilled water. After gently wiping off the water droplets and drying the chamber, the chamber was observed and photographed under a microscope.

### 2.11. Statistical Analysis

The results are expressed as the mean ± standard deviation (*x* ± *s*). All values were analyzed using SPSS 21.0 statistical software (IBM SPSS, USA), with *P* < 0.05 taken as statistically significant.

## 3. Results

### 3.1. Verification of Microarray Data by RT-qPCR

Five genes (*HOXD-AS2, HOXA11-AS, HOXA2, MMP7, and MMP9*) were randomly selected from the microarray data, and their levels of expression in the samples were detected by RT-qPCR. The log T/*N* value, which is the logarithm of the ratio of gene expression levels in tumor tissues and normal brain tissues, was calculated, and the result showed good consistency with the microarray result (Figure 1).

### 3.2. *HOXD-AS2* Is Highly Expressed in Glioma Tissue and Is Correlated with Poor Prognosis

As shown in Figure 2(a), the relative expression level of *HOXD-AS2/GAPDH* in tumor tissues of different grades was significantly higher than that in the normal brain tissue (*P* < 0.05). The relationship between the level of expression of the *HOXD-AS2* gene and the clinicopathological features of patients with glioma was analyzed. As shown in Table 3, it was found that the level of expression of the *HOXD-AS2* gene was only related to the pathological grade of the tumor (*P*=0.003).

According to the expression of the *HOXD-AS2* gene, 102 patients (the low-grade group included 45 patients with grade I–II glioma, and the high-grade group included 57 patients with grade III–IV glioma) were divided into a high-expression group and low-expression group. The Kaplan–Meier analysis and log-rank tests were performed to investigate the association between *HOXD-AS2* expression and the prognosis of the patients with glioma. It was found that the median survival time of the *HOXD-AS2* high-expression group was significantly shorter than that of the *HOXD-AS2* low-expression group (16 *vs.* 42 months, *P*=0.007, Figure 2(b)). Stratified analysis indicated that high expression of *HOXD-AS2* was significantly correlated with worse median survival time in patients with low-grade glioma (Figure 2(c)) but not in patients with high-grade glioma (Figure 2(d)), probably because of the small sample size of this subpopulation. Univariate analysis identified three prognostic factors: pathology grade (I–II or III–IV), extent of resection, and *HOXD-AS2* expression. Multivariate regression analysis of the prognosis factors confirmed that increased *HOXD-AS2* expression was an indicator of poor survival in glioma patients, in addition to pathology grade (*P* < 0.001) and extent of resection (*P*=0.026, Table 4).

### 3.3. Silencing of *HOXD-AS2* Expression in Glioma Cells

We subsequently measured the expression of *HOXD-AS2* in three glioma cell lines by real-time PCR. The expression level of *HOXD-AS2* was higher in U251 cells than in A172 and U87 cells, so we selected U251 cell lines for subsequent experimental studies (Figure 3(a)). To investigate the effect of *HOXD-AS2* knockdown on cell biological behavior, we used siRNA to inhibit its expression in glioma cells. Using the NC as the reference, SiHOXD-AS2-1 and SiHOXD-AS2-2 had greater interference efficacy, and therefore, SiHOXD-AS2-1 and SiHOXD-AS2-2 were selected as interference fragments in the subsequent cell function experiment (Figure 3(b)).

### 3.4. HOXD-AS2 Knockdown Inhibits U251 Cell Growth

The cell proliferation rate in the two interference groups was lower than that in the NC group, indicating that HOXD-AS2 gene knockdown affected cell proliferation ability (Figure 3(c)). We verified this result in the EdU incorporation assay. Interference fragments SiHOXD-AS2-1 and SiHOXD-AS2-2 were transfected into the U251 cell line. The number of cells in the NC group (U251 + Lipo 3000 + NC sequence) was used as the reference, and the nucleus was stained with EdU reagent. It was found that after 48 h of interference, the number of cells in the proliferative phase of the interference group was decreased; that is, the proportion of EdU-positive cells (red-stained nuclei in the figure) to the total number of cells (red-stained + blue-stained nuclei) was decreased (Figure 3(d)). In other words, the number of cells in the proliferative phase was decreased and the proliferative ability of cells was also decreased (SiHOXD-AS2-1 group *vs.* NC group, *P* < 0.001, SiHOXD-AS2-2 group *vs.* NC group, *P* < 0.05) in the interference group (Figure 3(e)).

We next analyzed the effect of *HOXD-AS2* knockdown on cell cycle distribution by PI staining and flow cytometry. It was found that after 48 h of interference, the number of cells in the proliferation phase (S phase + *G*2 phase) in the interference group was decreased (Figure 3(f)), indicating that the cell proliferation ability was weakened (S phase + *G*2 phase: SiHOXD-AS2-1 group *vs.* NC group, *P* < 0.001; SiHOXD-AS2-2 group *vs.* NC group, *P* < 0.001, Figure 3(g)).

### 3.5. *HOXD-AS2* Knockdown Shows No Significant Effects on U251 Cell Apoptosis

The percentage of dead cells, late apoptotic cells, surviving cells, and early apoptotic cells in the three cell groups was observed by flow cytometry to determine the effect of the *HOXD-AS2* gene on cell apoptosis (Figure 4(a)). The results showed that there was no significant change in the SiHOXD-AS2-1 group and the SiHOXD-AS2-2 group compared with the NC group (*P* > 0.05), indicating that HOXD-AS2 had no significant effect on apoptosis (Figure 4(b)).

### 3.6. Downregulation of *HOXD-AS2* Inhibits Glioma Cell Migration but Shows No Significant Effect on U251 Cell Invasion

To investigate further the function of *HOXD-AS2*, wound-healing assays were performed to measure the effect of *HOXD-AS2* knockdown on cell migration. The results showed that the migration ability of U251 cells was decreased significantly after interference *HOXD-AS2* (*P* < 0.001, Figures 5(a) and 5(b)). We also investigated whether *HOXD-AS2* affected the invasiveness of glioma cells. As shown in Figure 5, the cells in all three groups could pass through the matrix glue better (Figure 5(c)); that is, after interference with *HOXD-AS2*, the invasive ability of cells showed no significant change (*P* > 0.05, Figure 5(d)).

## 4. Discussion

Glioma is the most common primary tumor in the central nervous system, accounting for 80% of all malignant brain tumors [12]. At present, there is no very effective treatment for glioma, especially GBM. The average life expectancy of patients with GBM is only 4.5 months after diagnosis, although it can be extended to 15 months after surgery with temozolomide (TMZ) chemotherapy [13]. In addition, a large number of tumors may develop TMZ resistance, which seriously affects the clinical outcome of patients with GBM [14]. It is therefore essential to develop new and effective strategies for early diagnosis and treatment of glioma.

The *HOX* gene has been shown to be differentially expressed in many primary solid tumors, including breast cancer [15], lung cancer [16], cervical cancer [17], bladder cancer [18], melanoma [19], renal cell carcinoma [20], colon cancer [21], and prostate cancer [22]. Some *HOX* genes are also involved in translocations in cells in the hematopoietic system in malignant tumors [23]. It is reported that abnormal expression of *HOXB3*, *HOXB4,* and *HOXC6* is related to the formation of medulloblastoma and primitive neuroectodermal tumors in children [24, 25]. In addition, the *HOXD* gene is overexpressed in astrocytoma [26] and low-grade glioma in children [27]. Other studies suggest that *HOXD9* may be a molecular marker for glioma tumor stem cells, affecting the proliferation ability of glioma cells and the prognosis of patients with glioma [28]. Duan et al. [29] reported that the expression of *HOXA13* was related to the grade and prognosis of glioma. Bioinformatic analysis shows that most *HOXA13*-related genes are involved in cancer-related signal transduction pathways, especially in transcription regulation [30]. Cell proliferation, invasion, and apoptosis were decreased after overexpressing *HOXA13* in four glioma cell lines, and knocking down *HOXA13* expression inhibited the growth of in situ tumors [29]. Further study demonstrated that *HOXA13* partly promoted glioma progression through epithelial-mesenchymal transition induced by the *Wnt* and *TGF-β* pathways; this is known as a potential biomarker of GBM and an independent risk factor for prognosis in patients with advanced glioma [29].

The experiments in the above literature suggest that the *HOX* gene may be closely related to the occurrence and progression of glioma. In addition, lncRNA *HOTAIR* has been identified as an important marker of tumor grading and prognosis of glioma and is related to molecular subtypes in glioma [8]. Further study has found that *HOTAIR* interacted with and recruited *PRC2* to the *HOXD* site on chromosome 2, silencing transcription across the 40 kb region of *HOXD8*, *HOXD9*, H*OXD10,* and *HOXD11* on chromosome 2 [31, 32].

Based on the high expression of the *HOXD-AS2* gene in the chip data for five GBM tissue specimens *vs.* five normal brain tissue specimens, we aimed to explore the expression of *HOXD-AS2 (HOXD cluster antisense RNA 2)* in glioma and its relationship with the occurrence and progression of the malignancy. The expression of *HOXD-AS2* in normal brain tissue and in glioma tissues of different grades was detected by RT-qPCR. It was found that the expression of the *HOXD-AS2* gene was increased in glioma, and this tendency was positively correlated with the pathological grade of glioma. Survival analyses of patients with glioma in our experiment showed that expression of the *HOXD-AS2* gene was related to the prognosis of patients with glioma, especially those with low-grade glioma. The higher the expression of the *HOXD-AS2* gene, the worse the prognosis of the patients appeared to be.

To learn more about how *HOXD-AS2* genes play their role at the cytological level, we detected the expression of *HOXD-AS2* in U251, U87, and A172 cell lines and found that the expression of *HOXD-AS2* in U251 was the highest. Therefore, U251 cells were selected as the experimental cell line, and the expression of the *HOXD-AS2* gene in U251 cells was specifically knocked down by siRNA technology to observe its effect on U251 cell proliferation, invasion, apoptosis, and the cell cycle.

Using RNA interference technology, siRNA was used to knock down the expression of the *HOXD-AS2* gene specifically in glioma cell line U251, and we found that the proliferation and migration abilities of U251 cells were weakened, and the cell cycle was arrested. This result is consistent with the relationship between the level of expression of the *HOXD-AS2* gene and tumor grade and prognosis, demonstrating that glioma-related genes affected the prognosis of patients by affecting the biological characteristics of glioma cells. However, the specific molecular mechanism underlying this regulatory effect has not been fully studied in this study, and the particular mechanism by which HOXD-AS2 is upregulated in glioma is not clear. More studies are needed to verify the role of HOXD-AS2 as a reliable clinical predictor of the outcome for glioma patients in the future. Besides, we only did the interference experiment on the target gene, and the overexpression experiment was not carried out in this study, and it needs to be verified in other cell lines. In brief, it needs to be elucidated by further well-designed studies in the future.

## 5. Conclusion

*HOXD-AS2* is an oncogenic lncRNA associated with the poor prognosis of glioma. Knocking down the expression of *HOXD-AS2* can reduce the growth of glioma, which may provide a new strategy for the treatment of glioma. Our findings provide ideas for early diagnosis and treatment of glioma and possible strategies for improving the prognosis of glioma patients.

## Figures and Tables

**Figure 1:** Results of RT-qPCR showed good consistency with the microarray results.

**Figure 2:** Increased HOXD-AS2 expression confers poor prognosis in patients with glioma. (a) The relative expression values of *HOXD-AS2/GAPDH* in normal brain tissue and grade I, II, III, and IV gliomas were 0.0073 ± 0.0046, 0.0519 ± 0.0514, 1.3477 ± 2.2276, 1.9717 ± 2.9306, and 1.8884 ± 3.1063, respectively, showing significant differences between the normal brain tissue and tumor tissues of different grades (*P* < 0.05). (b) The Kaplan–Meier overall survival curves according to *HOXD-AS2* expression level. Glioma patients with high *HOXD-AS2* expression had significantly shorter median survival than patients with low *HOXD-AS2* expression (*P* < 0.001). (c, d) Low *HOXD-AS2* expression was significantly associated with longer median survival in patients with low-grade glioma (*P* < 0.05) but not in patients with high-grade glioma. NB, normal brain tissue; I–IV, I–IV glioma. ^*∗*^*P* < 0.05.

**Figure 3:** Levels of expression of HOXD-AS2 in U251 cell lines after siRNA transfection. Knockdown of HOXD-AS2 inhibits U251 cell growth. (a) The levels of expression of *HOXD-AS2* in three glioma cell lines were analyzed by RT-qPCR. (b) The levels of expression of *HOXD-AS2* in the U251 cell line were analyzed by RT-PCR; the relative gene expression level of SiHOXD-AS2-1—48 hr, SiHOXD-AS2-2—48 hr, and SiHOXD-AS2-3—48 hr was 0.20 ± 0.04, 0.34 ± 0.09, and 0.83 ± 0.12. NC, negative control; ^*∗∗*^*P* < 0.01. (c) Knockdown of *HOXD-AS2* reduced the growth of U251 cells compared with the NC group in the CCK-8 assay. (d) U251 cells were transfected with siRNAs, and after 48 h, cells were stained and imaged under a fluorescence microscope. Scale bars represent 50 *μ*m. (e) The ratio of EdU‐positive cells was calculated and plotted on the histogram. (f) Cell cycle profiling was analyzed using flow cytometry. The image shows the flow cytometry distribution of each cycle in the three groups of cells 48 h after transfection. (g) The proportion of cells in G1 phase in interference groups 1 and 2 was higher than that in the NC group, indicating that the number of cells in S phase and G2 phase was reduced significantly. Data were based on at least three independent experiments and shown as mean ± SD. ^*∗∗*^*P* < 0.01; ^*∗∗∗*^*P* < 0.001.

**Figure 4:** Detection of apoptosis by flow cytometry. (a) The percentage of dead cells (UL), late apoptotic cells (UR), surviving cells (LL), and early apoptotic cells (LR) in the three cell groups was observed by flow cytometry. (b) The proportion of phase 4 cells in the three cell groups did not change significantly. Data were based on at least three independent experiments and shown as mean ± SD. ^*∗*^*P* > 0.05.

**Figure 5:** Silencing of HOXD-AS2 inhibited cell migration in glioma cells. (a) Wound scratch assays were adopted to examine the migratory capacity. (b) The healing area in the SiHOXD-AS2-1 group and SiHOXD-AS2-2 group was significantly smaller than that in the NC group 36 and 72 h after scratching (^*∗∗∗*^*P* < 0.001). (c) The invasion ability of U251 cells from different groups was detected in Transwell assays. (d) The number of invasive cells in the SiHOXD-AS2-1 group and SiHOXD-AS2-2 group vs. the NC group. Data were based on at least three independent experiments and shown as mean ± SD. ^*∗*^*P* > 0.05.

**Table 1:** Reaction primers for RT-qPCR.

Gene name	Primer	Annealing temperature (C)	Product length (bp)
*GAPDH*	F: CGGATTTGGTCGTATTGGG R: CTGGAAGATGGTGATGGGATT	60	280

*HOXD-AS2*	F: CCTCAGAAGCCCAGAAGAC R: GCCCTCATTCCCCAAGTTG	60	123

*HOXA11-AS*	F: CGGCTAACAAGGAGATTTGG R: CGTAAGGCTCAGGGATGGTA	60	257

*HOXA2*	F: TGGGAGCCTCGTCTCCTGGA R: TTGCTTCACATAAGTTTGGCTGGA	60	181

*CCNB2*	F: GATGAACTGGCGAGAGGTCTG R:TTTCAAACACCCACATTTCAACCC	60	157

*SOX2OT*	F: GGCTGGGCTTGGGCTTTATC R: AAGAAGGAAAGGGCACACTTGG	60	210

*MMP7*	F: GCCACCTGTAGGAATTAGAAGAC R: ATTCATCCGAGTGTTAGCAG	60	98

**Table 2:** Three interference sequences and NC sequence.

Number	Gene name	Sequence (5′-3′)
SiHOXD-AS2-1	*HOXD-AS2-homo-584*	**Sense (5′-3′)**: CCCAAGGAUUCAGCAAACATT
		**Antisense (5′-3′)**: UGUUUGCUGAAUCCUUGGGTT

SiHOXD-AS2-2	*HOXD-AS2-homo-633*	**Sense (5′-3′)**: GGAUGUGAAAUAGCACUUCTT
		**Antisense (5′-3′)**:GAAGUGCUAUUUCACAUCCTT

SiHOXD-AS2-3	*HOXD-AS2-homo-136*	**Sense (5′-3′)**:CGUCUGCUGUAAUCCACUATT
		**Antisense (5′-3′)**:UAGUGGAUUACAGCAGACGTT

NC		**Sense (5′-3′)**: UUCUCCGAACGUGUCACGUTT
		**Antisense (5′-3′)**: ACGUGACACGUUCGGAGAATT

**Table 3:** Correlations between the expression of *HOXD-AS2* and clinicopathologic parameters.

Parameter	Patients (n)	Expression of HOXD-AS2 (n)			*P* value
		Low (*n*, %)	Middle (*n*, %)	High (*n*, %)	
Total	87	29 (33.3%)	29 (33.3%)	29 (33.3%)	
Age					
<55	52	22 (42.3%)	13 (25.0%)	17 (32.7%)	0.054
≥55	35	7 (20.0%)	16 (45.7%)	12 (34.3%)	
Gender					
Male	48	15 (31.3%)	16 (33.3%)	17 (35.4%)	0.870
Female	39	14 (35.9%)	13 (33.3%)	12 (30.8%)	
Tumor size					
<5 cm	30	14 (46.7%)	9 (30.0%)	7 (23.3%)	0.137
≥5 cm	57	15 (26.3%)	20 (35.1%)	22 (38.6%)	
Resection					
Total	52	22 (42.3%)	17 (32.7%)	13 (25.0%)	0.140
Subtotal	29	5 (17.2%)	11 (37.9%)	13 (44.8%)	
Partial	6	2 (33.3%)	1 (16.7%)	3 (50.0%)	
Pathology					
Low grade	40	20 (50.0%)	7 (17.5%)	13 (32.5%)	0.003
High grade	47	9 (19.1%)	22 (46.8%)	16 (34.0%)	

**Table 4:** Analysis of different prognostic factors in patients with glioma.

Variables	Univariate HR (95% CI)	*P* value	Multivariate HR (95% CI)	*P* value
Age	2.53 (1.33–4.80)	0.004	1.65 (0.82–3.33)	0.165
Gender	1.38 (0.75–2.53)	0.304	1.67 (0.87–3.19)	0.123
Pathology grade	4.61 (2.27–9.37)	<0.001	4.27 (1.89–9.65)	<0.001
Tumor size	1.37 (0.71–2.67)	0.351	1.22 (0.62–2.41)	0.563
Extent of resection	1.55 (1.01–2.37)	0.043	1.82 (1.07–3.09)	0.026
*HOXD-AS2* expression	2.33 (1.22–4.43)	0.01	1.31 (0.66–2.61)	0.448

## Data Availability

The data used to support the findings of this study are included within the article.
